This article has been retracted.

# Evaluation of Live Recombinant Nonpathogenic *Leishmania tarentolae* Expressing Cysteine Proteinase and *A2* Genes as a Candidate Vaccine against Experimental Canine Visceral Leishmaniasis

**DOI:** 10.1371/journal.pone.0132794

**Published:** 2015-07-21

**Authors:** Mehdi Shahbazi, Farnaz Zahedifard, Tahereh Taheri, Yasaman Taslimi, Shahram Jamshidi, Sadegh Shirian, Niousha Mahdavi, Mehdi Hassankhani, Yahya Daneshbod, Sayyed Hamid Zarkesh-Esfahani, Barbara Papadopoulou, Sima Rafati

**Affiliations:** 1 Department of Immunotherapy and *Leishmania* Vaccine Research, Pasteur Institute of Iran, 69 Pasteur Ave., Tehran, 13164, Iran; 2 Department of Immunology, School of Medicine, Isfahan University of Medical Sciences, Isfahan, Iran; 3 Department of Internal Medicine, Faculty of Veterinary Medicine, University of Tehran, Tehran, Iran; 4 Department of Molecular and Cytopathology, Daneshbod Pathology Laboratory, Shiraz, Iran; 5 Research Center in Infectious Diseases, CHU de Québec Research Center and Department of Microbiology, Infectious Disease and Immunology, Laval University, Quebec, QC, Canada; London School of Hygiene and Tropical Medicine, UNITED KINGDOM

## Abstract

Canine Visceral Leishmaniasis (CVL) is a major veterinary and public health problem caused by *Leishmania infantum* (*L*. *infantum*) in many endemic countries. It is a severe chronic disease with generalized parasite spread to the reticuloendothelial system, such as spleen, liver and bone marrow and is often fatal when left untreated. Control of VL in dogs would dramatically decrease infection pressure of *L*. *infantum* for humans, since dogs are the main domestic reservoir. In the past decade, various subunits and DNA antigens have been identified as potential vaccine candidates in experimental animal models, but none has been approved for human use so far. In this study, we vaccinated outbreed dogs with a prime-boost regimen based on recombinant *L*. *tarentolae* expressing the *L*. *donovani* A2 antigen along with cysteine proteinase genes (CPA and CPB without its unusual C-terminal extension (CPB^-CTE^) and evaluated its immunogenicity and protective immunity against *L*. *infantum* infectious challenge. We showed that vaccinated animals produced significantly higher levels of IgG2, but not IgG1, and also IFN-γ and TNF-α, but low IL-10 levels, before and after challenge as compared to control animals. Protection in dogs was also correlated with a strong DTH response and low parasite burden in the vaccinated group. Altogether, immunization with recombinant *L*. *tarentolae* A2-CPA-CPB^-CTE^ was proven to be immunogenic and induced partial protection in dogs, hence representing a promising live vaccine candidate against CVL.

## Introduction

*Leishmania infantum* is the causative agent of both canine leishmaniasis and zoonotic visceral leishmaniasis in children and immune-compromised adults. In humans as well as dogs, disease symptoms are severe and can be fatal if left untreated. The dog is the major reservoir of *L*. *infantum* in the Middle East and the Mediterranean region and of *L*. *donovani chagasi* in South America. The pattern of the disease in dogs and humans is similar and both of them show long period of asymptomatic infection [1]. In addition, the outcome of disease in dogs is variable and infection is not equal to disease.

An estimated of 200,000 to 400,000 new cases (http://www.who.int/mediacenter/factsheets/fs375/en) have been diagnosed with VL worldwide, and there are reports of a dramatic increase in the number of human leishmaniasis [2] and also of VL-HIV-1 co-infection in endemic areas [3]. Control of the disease mainly depends on chemotherapy, which is too expensive with extensive toxicity complications. In addition, in some cases chemotherapy leads to the development of resistant parasites [4]. Treatment of infected dogs will often achieve clinical remission, relapses are reported to occur frequently and the animals remain infectious to the vector [5, 6]. Therefore, much attention has been given to the development of effective vaccines. Leishmanization or inoculation of virulent *Leishmania* is the oldest vaccination strategy against cutaneous leishmaniasis (CL) and recently against VL [2, 7]. Although leishmanization has shown improved long-term immunity and recovery of individuals from CL resisted reinfection, a variety of adverse effects has been observed, including the development of large persistent lesions and psoriasis [2]. During the past several decades, different formulations have been examined to devise an effective *Leishmania* vaccine, including killed, live attenuated parasites, recombinant *Leishmania* proteins or DNA encoding *Leishmania* proteins [3, 8]. To date, several vaccination strategies have been tried against experimental leishmaniasis, and most of them emphasize on CL rather than VL [9].

Previous studies have shown that the presence of small parasite numbers seems to be required for the development of *Leishmania*-specific effector cells and maintenance of anti-*Leishmania* immunity [10, 11]. For this purpose, the use of live attenuated organisms is an attractive strategy for vaccination and thus more recent experimentations have led to the development of attenuated strains that mimic more closely the natural course of infection [12–14]. However, this type of vaccines has also its limitations such as a risk of reverting to virulence, liability of production in the large scale and distribution in the field [9]. Although parasite persistence is necessary for the maintenance of effector T cells, it has been shown that central memory T cells (CD62L^high^, IL-2^pos^, IFN-γ^neg^) could develop in the absence of parasites [13]. A new approach has been introduced by Breton *et al*. using a non-pathogenic to humans *Leishmania* (*L*. *tarentolae*) as an experimental vaccine against VL [15]. *L*. *tarentolae* can differentiate into amastigote forms but is unable to survive long enough within mammalian macrophages and to establish disease. Moreover, *L*. *tarentolae* activates dendritic cell maturation, induces T-cell proliferation and the production of IFN-γ [15]. Our previous study in mice has established the use of recombinant *L*. *tarentolae* expressing the *L*. *donovani* A2 antigen along with cysteine proteinases (CPA and CPB^–CTE^) as a safe and promising vaccination strategy against VL [16]. Since the pattern of VL in dogs and humans is similar [1], dogs represent the best animal model for evaluating protective immune responses of candidate vaccines against visceral leishmaniasis [9].

In recent years, several antigens have been examined as candidate vaccines in dogs, including FML [17–19], *Li*ESA [20, 21], P8 [22], rA2 [23], protein Q [24], rTSA, rLeIF and LmSTI1 [25], rMML [26], rORFF [27], LACK [28] and cysteine proteinases (CPs) type I and II [29]. Furthermore, the FML-saponin vaccine under the name of Leishmune [19], and the recombinant A2-antigen adjuvanted by saponin called LeishTec [23] were licensed for prophylaxis against canine ZVL and has been used in Brazil, and also a formulation related to the *Li*ESAp vaccine was licensed for commercialization under the name of CaniLeish [30, 31] in Europe.

We have shown previously that prime and boost immunization with A2-CPA-CPB^-CTE^ recombinant *L*. *tarentolae* protects BALB/c mice against *L*. *infantum* challenge and that protection was associated with high levels of IFN-γ, lower levels of IL-10, high nitric oxide production and low parasite burden [16]. In this study, we evaluated the immunogenicity and protective immunity of recombinant *L*. *tarentolae* expressing A2-CPA-CPB^-CTE^ as a live vaccine against VL in dogs. Recombinant *L*. *tarentolae* was administered subcutaneously both as prime and boost regimen. Vaccinated dogs were followed for almost 20 months and different parameters, including cellular and humoral immune responses, parasite load in bone marrow, and clinical evaluations revealed a partial protection against an infectious *L*. *infantum* challenge.

## Materials and Methods

### Ethical consideration

All procedures including maintenance, animals’ handling program, blood and bone marrow sample collection were approved by Institutional Animal Care and Research Advisory Committee of Pasteur Institute of Iran (Grant ID 564 dated 2011) and Veterinary Board of Tehran Medical school (700/4038 dated 2011) based on the specific National Ethical Guidelines for Biomedical Research issued by the Research and Technology Deputy of Ministry of Health and Medicinal Education (MOHME) of Iran (2005).

### Parasites

Live *L*. *tarentolae* harboring A2 and CPs genes were generated in our previous study [16]. The *L*. *tarentolae* wild type strain and recombinant *L*. *tarentolae* A2-CPA-CPB^-CTE^ were grown in M199 medium supplemented with 5% heat-inactivated fetal calf serum, 40 mM HEPES (pH 7.2), and 50 μg/ml gentamicin at 26°C. The *L*. *infantum* strain MCAN/ES/98/LLM-877 was kindly provided by the WHO collaborating center for leishmaniasis, Servicio de Parasitología, Centro Nacional de Microbiología, Instituto de Salud Carlos III, Madrid, Spain and was kept virulent by continuous passage in hamsters. Stationary phase *L*. *infantum* promastigotes were used for infectious challenge grown at 26°C in Novy-MacNeal-Nicolle (NNN) medium supplemented with 10% heat-inactivated FCS, 40 mM HEPES, 0.1 mM adenosine, 0.5 μg/ml hemin and 50 μg/ml gentamicin.

### Animals

Three groups of dogs were allocated for this experiment. Thirty healthy mixed breed dogs (18 males and 12 females and weight 19 ± 4 kg) were selected from a non-endemic part of Iran (Tehran and Mashhad cities). Prior to the beginning of the trial (2 months in advance), not only all dogs were vaccinated for distemper (DHP produced by NOBIVAC, Intervet), canine parvovirus (CPV strain 154), canine adenovirus (CAV 2 strain Manhatan LPV3) and rabies (BHK, produced by Pasteur Institute of Iran), but also they received an oral anti-helminthic treatment. Prior to vaccination, blood was collected and then sera and genomic DNA of all dogs were separated and extracted in order to exclude any infected dog or possible exposure to *Leishmania*. All dogs had a specific code/ID throughout the experiment. Dogs were between 6 months to 4 years old (the age of dogs was determined based on changes of tooth color, tartar building-up, reduce tooth wear and gum inflammation as recommended by Animal sheltering (WWW.ruralareavet.org). Dogs were housed individually in conventional kennels (90*110*170cm) at the School of Veterinary Medicine, Tehran University and fed with standard commercial diet (Nutripet, Iran). Animals were acclimated for three/four months in the animal facility and temperature (15–20°C), light/dark (12h on/12h off), humidity (40–60%) and food were controlled every day. During the whole period of our study (every day) the welfare including separate cage with soft floor mat, optimum temperature and humidity, free access to water and once per day access to food were strictly applied. In addition, all dogs had daily access to the outside about 30 min. The conditions of the animals were followed by veterinarians routinely (including appetite, physical examination and physical activity) and every 3 months CBC and serum biochemistry tests were measured. All the invasive procedures were performed following the rules of ethical procedures in animal experimentation and biosafety.

### Vaccine administration and experimental infection

Dogs were divided into three groups (according to their weight, sex and age, each including 10 dogs) named as G1, G2 and G3. The first group (G1) was immunized subcutaneously (SC) with 2x10^7^ *L*. *tarentolae* A2-CPA-CPB^-CTE^ EGFP. Group G2 was immunized with wild type (WT) *L*. *tarentolae* and G3 was immunized with PBS. Three weeks later, all groups were immunized similarly as booster. Three weeks after boost, all groups were challenged by intravenous injection with 4 x 10^7^ *L*. *infantum* (MCAN/ES/98/LLM-877) stationary phase promastigotes.

### Evaluation of humoral immune response

Sera of dogs were collected at different time courses (T0: before challenge at day 41; T1: 2 months after challenge at day 60; T2: 6 months after challenge at day 180; T3: 11 months after challenge at day 330; T4: 14 months after challenge at day 420; T5: 17 months after challenge at day 510) in order to measure individually the level of specific antibody production against freezed/thawed *L*. *tarentolae* A2-CPA-CPB^-CTE^-EGFP and freezed/thawed *L*. *infantum* crude lysate. Briefly, similar to our previous studies [29], the plates were incubated overnight at 4°C and then blocked with 1% (w/v) BSA in PBS at 37°C for 2 h. Sera were diluted and added at 1:100 in PBS supplemented with 0.05% (v/v) Tween 20 and 1% (w/v) BSA. After incubation for 2 h at 37°C, plates were washed three times with PBS containing 0.05% (v/v) Tween 20, then goat anti-dog IgG1 (Bethyl Laboratories Inc., Montgomery, TX, USA) and sheep anti-dog IgG2 (Bethyl Laboratories Inc., Montgomery, TX, USA) conjugated to peroxidase were used and incubated for 2 h at 37°C. IgG1 and IgG2 conjugates were diluted in PBS–0.05% (v/v) Tween 20–1% (w/v) BSA at 1:10,000 and 1:50,000, respectively. The plates were washed three times and binding of conjugate was visualized with Peroxidase substrate system (KPL, ABTS). The reaction was stopped by adding 1% SDS and absorbance value was measured at 405 nm in an automatic micro-ELISA reader. In all tests, sera from infected dogs were used as a positive control and sera from healthy dogs as a negative control.

### Evaluation of cytokine production

Levels of IFN-γ, TNF-α and IL-10 were assessed before (T0) and two (T1), six (T2), eleven (T3), fourteen (T4) and seventeen (T5) months after challenge. For this purpose, peripheral blood mononuclear cells (PBMCs) were obtained from heparinized blood, mixed 1:1 with PBS at room temperature, layered over Ficoll (Histopaque 1077 Sigma, USA) and centrifuged at 2200 rpm for 30 min at room temperature. PBMCs were collected and then washed twice in DMEM medium (centrifuged at 1700 rpm, for 10 min). The pelleted cells were resuspended in 1 ml DMEM medium and cells were counted with a haemocytometer. The isolated PBMCs were resuspended in DMEM medium supplemented with 20% (v/v) heat-inactivated FCS, 10 mM HEPES, and 50 μg/ml gentamicin. 1.5 ml of cell suspension (3×10^6^ /ml) was plated in duplicated 48-well culture plates. Isolated PBMCs were incubated for 96 h in the presence of 10 μg/ml of PHA (as positive control), 20 μg/ml of *L*. *tarentolae* A2-CPA-CPB^-CTE^-EGFP (F/T), and 20 μg/ml of *L*. *infantum* (F/T) or in the absence of antigens (as negative control) at 37°C and 5% CO_2_. The supernatants were collected for assessing the production of IL-10 and TNF-α after 24 h, for IFN-γ after 96 h, then stored at -70°C until assayed by the sandwich ELISA (Duoset ELISA Canine IFN-γ, Duoset ELISA canine TNF-α and Duoset ELISA canine IL-10; R&D Systems). For the assay, specific mouse anti-dog IFN-γ (1 μg/ml), mouse anti-dog IL-10 (2 μg/ml) and mouse anti-dog TNF-α (2 μg/ml) antibodies as the capture antibody and biotinylated goat anti-dog IFN-γ (4 μg/ml) and goat anti-dog IL-10 (100 ng/ml), goat anti-dog TNF-α (100 ng/ml) antibodies as the detection antibody were used. The test was developed with ABTS 2-Component Microwell Peroxidase Substrate system kit. The reaction was stopped by 1% SDS and the absorbance value was measured at 405 nm in an automatic micro-ELISA reader. Standard curves for IFN-, TNF-α and IL-10, respectively, were performed by the use of recombinant canine proteins. Detection limits were 17.5–2000 pg/ml for the canine IFN-γ and IL-10 and also 8.75–1000 pg/ml for TNF-α, according to the manufacturer kits.

### Leishmanin skin test

The delayed type hypersensitivity (DTH) was determined by intradermal injection, at 11 and 16 months after challenge. Dogs were inoculated intradermally in the right shaved groin with 3×10^8^/ml stationary phase promastigotes of *L*. *infantum* in 0.4% phenol-saline [32]. The left shaved groin received only 0.1 ml saline (control). The largest diameter of the induced indurations and their perpendicular diameter were measured at 48 hours. Indurate areas were marked, and each time the values of the saline control were subtracted from the reaction due to the *Leishmania* antigen. Reactions showing diameters ≥5mm were considered positive.

### Real time PCR in bone marrow

Bone marrows from all dogs were taken at 18 months after challenge. Dogs were anesthetized with a mixture of medetomidine hydrocholoride (Domitor) and ketamine (5 mg/kg). The bone marrow was aspirated from the iliac bone with a 16 mm x 25 mm Klima needle into 20 ml syringe containing 0.5% EDTA in RPMI. Each sample was divided into three parts for quantification of parasite burden by using cytology, immunocytochemistry (ICC), and real time PCR examinations. Real time PCR was used to quantify the parasite load in the bone marrow 18 months post-challenge. One milliliter of bone marrow iliac aspirates were collected into EDTA tubes and stored at −20°C. Genomic DNA was extracted from 200 μl of bone marrow using DNeasy Blood & Tissue kit (Qiagen). Two sets of primers which targeting a region of kinetoplastid minicircle DNA of *L*. *infantum* named as RV1 and RV2 (forward:-CTTTTCTGGTCCCGCGGGTAGG-39; reverse: 59-CCACCTGGCCTATTTTACACCA-39) were used [33]. Quantification of *Leishmania* DNA was performed using an absolute method, by comparison of Ct values with those from a standard curve constructed from 10-fold dilutions of *L*. *infantum* DNA extracted from cultured parasites, from 1×10^6^ to 0.1 parasite equivalents/ml, using Applied Biosystem 7500 real time PCR system. All samples were run in duplicates on every plate. For quantification of parasites in bone marrow, 200 ng of DNA was subjected to the reaction containing 5 pmol of each forward and reverse primers, 12.5 μl Qiagen QuantiFast SYBR Green Master Mix in total volume of 25 μl. Conditions for PCR amplification were as follows: 95°C for 10 min; 40 cycles consisting of 95°C for 15 s, 58°C for 30 s, and 72°C for 40 s. Specific amplification of the target region was confirmed by gel electrophoresis of the PCR products.

### Cytology and immunocytochemistry (ICC)

Multiple aspirated smears were made on slides and were both air-dried and alcohol-fixed and stained by Wright and Giemsa methods. Specific antibody (WHO LXXVIII-2E5-A8 (D2) for *L*. *donovani/L*. *infantum* used as a primary antibody that was available from our previous study [34]. The slides were rehydrated and treated with 3% hydrogen peroxide solution for 10 minutes at room temperature to quench endogenous peroxides. The antigen retrieval was conducted by pre-treatment with microwaving (power 100 for 10 min and then power 20 for 20 min) using a 10-mmol/L concentration of citrate buffer (pH 6.0) and proteinase K. The primary antibody was applied for 1 hour (diluted 1:200). Detection of the immunoreaction was achieved. The detection system used was Envision+ (DakoCytomation) and developed with diaminobenzidine (Dako Cytomation). 3, 3’-diaminobenzidine-hydrogen peroxide was applied as the chromogen and hematoxylin was used as the counterstain. The cytological and immunocytochemistical smears were examined under different magnifications. The modified scoring method, explained by Shirian *et al*. [35], was used for leishman body burden. The samples were considered negative if amastigotes were not found in 1000X magnification (oil immersion field, OIF) in the whole slide smear. The density of amastigotes was quantified using a semi-quantitative scale according to Table 1.

**Table 1:** Cytological and immunocytochemical diagnosis of vaccinated and unvaccinated dogs experimentally infected with *L*. *infantum*.

No. Case	Cytology	Immunocytochemistry
**Group 1(G1)**		
2	++	++
4	++	+
6	+	+
12	+	++
13	++	++
19	++	++
24	++	+
25	+	++
48	++	++
**Group 2(G2)**		
16	++	++
17	+	++
31	+++	+++
34	++	++
41	++	++
42	+	+
44	++++	++++
65	+	+
**Group3 (G3)**		
7	+	+
11	++++	++++
20	++	++
43	+	+
45	+++	+++
47	+++	+++
49	++	++
50	++++	++++
62	++++	++++

Grade I (+): mean 5–10 leishman bodies in 40 oil immersion field (OIF).

Grade II (++): mean 10–20 leishman bodies in 30 OIF.

Grade III (+++): mean 20–50 leishman bodies in 20 OIF.

Grade IV (++++): more than 50 leishman bodies in 10 OIF

### Endpoint culture of spleen tissues

All dogs were sacrificed by intravenous injection of thiopental sodium 33% (5 ml/kg) at the end of the study (20 months post-infection). A piece of spleen was removed in aseptic conditions and cultured in 2 ml of Schneider’s *Drosophila* medium supplemented with 20% heat-inactivated fetal calf serum and gentamicin (0.1%). After incubation at 26°C, the cultures were examined daily for the presence of promastigotes under an inverted microscope at a magnification of 40X during 1 month periods.

### Clinical examination and biochemical evaluations

Routine clinical evaluation of the animals was carried out every 3 months. In each evaluation, dogs were weighed and their general health status was examined by a veterinarian. At the end of project, all dogs were clinically classified, according to presence/absence of infection signs: subpatent (clinically well and bone marrow DNA positive only), asymptomatic (clinically well, bone marrow DNA positive and spleen culture positive), or symptomatic when the dogs showed one or more clinical signs of CVL including, lymphadenopathy, alopecia, weight loss, bone marrow DNA positive and also spleen culture positive [36, 37]. Biochemical analysis was performed in all animals 20 months after challenge. Serum levels of alanine aminotransferase (ALT), aspartate aminotransferase (AST), urea, creatinine, alkaline phosphatase (ALP), albumin(Alb) and total proteins were determined by a biochemistry serum analyzer (Technicon RA-1000, USA).

### Statistical analysis

Statistical analyses were performed using Graph-Pad Prism 5.0 for Windows (Graphpad Software Inc 2007, San Diego, USA) as well as SPSS version 18. Data were expressed as median. Each group (G1 and G2) were compared with control PBS group (G3). In some cases, G1 and G2 were compared similarly. Non-parametric analysis were used for all tests including humoral, cellular immune responses, DTH responses and parasite load since they were not normally distributed. Mann—Whitney test and Fishers exact test were also used for the comparison of different parameters between groups. The correlation between the IFN-γ and IgG2 production at 14 and 17 months after challenge was calculated using Spearman correlation method for each group (G1, G2 and G3). The *p* value <0.05 was considered significant.

## Results

### Vaccination regimens and clinical follow up

To assess the ability of recombinant *L*. *tarentolae* A2-CPA-CPB^-CTE^-EGFP to protect dogs against challenge with *L*. *infantum*, 30 outbreed dogs subdivided into three groups (G1 to G3) were tested. The first group (G1) was vaccinated subcutaneously with two doses of *L*. *tarentolae* A2-CPA-CPB^-CTE^-EGFP, the second group (G2) received two doses of *L*. *tarentolae* wild type (WT), and the third group (G3) received two doses of PBS alone and used as a control. Additional details about the route of vaccination, dose interval, and vaccine formulation are summarized in Table 2. Animals were followed up throughout the duration of the experiment for 20 months to evaluate clinical symptoms of leishmaniasis, as well as the development of cellular and humoral immune responses (S1 Fig). The vaccine was well tolerated and there was no local reactivity at the point of inoculation. One dog from each group died during the study for reasons unrelated to canine leishmaniasis (gastric dilatation volvulus (GVD) and Uremia and Chronic kidney disease). In addition, one animal from G2 (16 months post-infection) and one from G3 (20 months post-infection) died from visceral leishmaniasis.

**Table 2:** Vaccination regimens in different dog groups. The first group (G1) was immunized subcutaneously (*sc*) with 2x10^7^ *L*. *tar*A2-CPA-CPB^-CTE^ GFP (recombinant (r) rLive/rLive). The second group (G2) was immunized *sc* with *L*. *tarentolae* (WT) and the third group (G3) was injected with PBS. Three weeks after priming, all groups were boosted similarly. Three weeks after the boost, all groups were challenged by intravenous (*iv*) injection of 4 x 10^7^ *L*. *infantum* metacyclic promastigotes. PBS: Phosphate saline buffer.

Groups	Priming (day 0)	Boosting (day 21)	Challenge (day 42)	Modality
**Group 1 (N = 10)**	*L*. *tarentolae*A2-CPA-CPB^-CTE^-EGFP (*sc*)	*L*. *tarentolae*A2-CPA-CPB^-CTE^-EGFP (*sc*)	*L*. *infantum* (*iv*)	rLive/rLive
**Group 2 (N = 10)**	*L*. *tarentolae* (WT) (*sc*)	*L*. *tarentolae*(WT) (*sc*)	*L*. *infantum* (*iv*)	rLive/rLive
**Group 3(N = 10)**	PBS (*sc*)	PBS (*sc*)	*L*. *infantum* (*iv*)	Control

### Antibody responses to leishmanial antigens

Specific IgG1 and IgG2 antibodies against *L*. *infantum* and *L*. *tarentolae* A2-CPA-CPB^-CTE^-EGFP (F/T) were measured in the sera of all dogs by ELISA. At the starting point, before challenge (T0, day 41), sera reactivity was measured only against *L*. *tarentolae* A2-CPA-CPB^-CTE^-EGFP and for the rest of the time points, including 3(T1), 7(T2), 12(T3), 15(T4) and 18(T5) months post-challenge both *L*. *tarentolae* A2-CPA-CPB^-CTE^-EGFP and *L*. *infantum* (F/T) were considered. The results are presented in Fig 1. Levels of anti-*L*. *infantum* (F/T) IgG1 antibody were increased after challenge (Fig 1A). Group 3 showed significantly higher levels of anti-*L*. *infantum* IgG1 at T2, T3 and T5 compared to G1 (*p*<0.001, *p*<0.001 and *p*<0.05, respectively) and also at T2 and T3 in comparison to G2 (*p*<0.05). Interestingly, the levels of IgG1 at T4 in G2 were significantly higher than in G1 and G3 for the same period (*p*< 0.05). The specific levels of IgG2 against *L*. *infantum* (F/T) were significantly higher in G1 compared to the control group (G3) at T5 (*p*<0.05). Similarly in G2, the most significant difference was observed at T3-T5 (*p*<0.01, *p*<0.01 and *p*<0.05, respectively) as compared to PBS group (G3) (Fig 1B).

**Fig 1:** Analysis of specific humoral response elicited in vaccinated and controls groups. Serum from all dogs was obtained at different time points throughout the experiment. T0: before challenge at day 41; T1: 2 months after challenge at day 60; T2: 6 months after challenge at day 180; T3: 11 months after challenge at day 330; T4: 14 months after challenge at day 420; T5: 17 months after challenge at day 510. Anti-*L*. *infantum* (F/T) IgG1 (A), anti-*L*. *infantum* IgG2 (B) and anti-*L*. *tarentolae* A2-CPA-CPB^-CTE^-EGFP (F/T) IgG1 (C), anti-*L*. *tarentolae* A2-CPA-CPB^-CTE^-EGFP (F/T) IgG2 (D), IgG2/IgG1 ratio against *L*. *infantum* (F/T) (E) and IgG2/IgG1 ratio *L*. *tarentolae* A2-CPA-CPB^-CTE^-EGFP (F/T)(F) production were determined by ELISA. The asterisk indicates the significant difference between values at the indicated time points as determined by Student’s test (*p*< 0.05 denoted as *, *p*<0.01 denoted as **, *p*<0.001 denoted as *** and n.s. denoted as non significant).

Significantly higher levels of specific IgG1 against *L*. *tarentolae* A2-CPA-CPB^-CTE^-EGFP (F/T) were detected in G3 at T2 and T3 than in G1 (*p*<0.01 and *p*<0.05, respectively) and only at T0 for G2 (*p*<0.05) (Fig 1C). Levels of IgG2 against *L*. *tarentolae* A2-CPA-CPB^-CTE^-EGFP (F/T) in G1 and G2 were significantly higher than G3 at T0-T3 (*p*<0.05) (Fig 1D).

IgG2/IgG1 ratios in respect to *L*. *infantum* (F/T) are shown in Fig 1E. The IgG2/IgG1 ratio in G1 was significantly higher than in G3 for the periods T3-T5 *(p*<0.001, *p*<0.05 and *p*<0.001, respectively) and in G2 at T3 and T5 (*p*<0.001 and *p*<0.05, respectively). The IgG2/IgG1 ratio in the G1 and G2 against *L*. *tarentolae* A2-CPA-CPB^-CTE^-EGFP (F/T) was significantly higher than in G3 for periods T0,T2 and T3 (*p*<0.05, *p*<0.01 and *p*<0.01 for G1; *p*<0.05, *p*<0.05 and *p*<0.05 for G2, respectively) as shown in Fig 1F. Overall, our data indicate that humoral response (IgG2) in the vaccinated group (G1) was significantly higher than in the control group (G3).

### Measurement of IFN-γ, TNF-α and IL-10 production in PBMCs

Different cytokines including IFN-γ, TNF-α and IL-10 were measured following stimulation with *L*. *infantum* (F/T) antigen in PBMCs at different time intervals as shown in Fig 2. The levels of IFN-γ at T1, T4 and T5 in G1 (*p*<0.05, *p*<0.01 and *p*<0.05, respectively) and in G2 only at T4 (*p*< 0.05) were significantly higher than in the G3 control group (Fig 2A).

**Fig 2:** Assessment of IFN-γ, TNF-α and IL-10 levels in PBMCs. Panel (A) shows IFN-γ levels detected after challenge in PBMC culture supernatants stimulated with *L*. *infantum* (F/T) at different time points post-infection. Panel (B) shows levels of IFN-γ detected in PBMC culture supernatants produced in response to *L*. *tarentolae* A2-CPA-CPB^-CTE^-EGFP (F/T) before challenge and at different time points post-infection. Panel (C) shows the levels of IL-10 in response to *L*. *infantum* (F/T) at different time points after infection. Panel (D) shows levels of IL-10 in response to *L*. *tarentolae* A2-CPA-CPB^-CTE^-EGFP (F/T) before challenge and at different time points after infection. Panel (E) shows IFN-γ/IL-10 ratio in response to *L*. *infantum* (F/T) at different time points. Panel (F) shows IFN-γ/IL-10 ratio in response to *L*. *tarentolae* A2-CPA-CPB^-CTE^-EGFP (F/T) before challenge and at different time points after infection. Panel (G) shows levels of TNF-α in response to *L*. *infantum* (F/T) at different time points after infection. Panel (H) shows levels of TNF-α in response to *L*. *tarentolae* A2-CPA-CPB^-CTE^-EGFP (F/T) before and at different time points after infection. The asterisk indicates the significant difference between values at the indicated time points as determined by Student’s test (p< 0.05 denoted as *, p<0.01 denoted as **, p<0.001 denoted as *** and n.s. denoted as non significant).

In response to *L*. *tarentolae* A2-CPA-CPB^-CTE^-EGFP (F/T), the level of IFN-γ in G1 was increased at T0-T5, and significantly higher levels were observed in G3 (*p*<0.01, *p*<0.001, *p*<0.001, *p*<0.05, *p*<0.05 and *p*<0.05 for each time intervals, respectively). We only observed a significant difference in IFN-γ production between G2 and G3 at T0-T2 (*p*<0.01, *p*<0.01and *p*<0.001 for each time intervals, respectively) (Fig 2B).

Following stimulation with *L*. *infantum* (F/T), we observed a remarkable increase in IL-10 levels in G3 at T1-T5 intervals (*p*<0.05) in comparison to the G1 group but at T2 only a significant difference (*p*<0.05) between G2 and G3 was observed (Fig 2C). As shown in Fig 2D, IL-10 production in response to *L*. *tarentolae* A2-CPA-CPB^-CTE^-EGFP was significantly higher in G3 than in G1 at different time intervals including T1, T2, T3 and T5 (*p*< 0.001, *p*<0.01, *p*<0.05 and *p*<0.05 for each time intervals, respectively) and only at T1 in G2 (*p*<0.05).

We further calculated the IFN-γ to IL-10 ratio for each dog as a clear indicator of successful immunization and protection levels [38]. As shown in Fig 2E, there were significant ratio differences between G1 and G3 at T3-T5 in response to *L*. *infantum* (F/T) (*p*<0.05, *p*<0.01 and *p*<0.001 for each time interval, respectively) and only at T4 (*p*<0.05) between G2 and G3. The IFN-γ/IL-10 ratio in response to *L*. *tarentolae* A2-CPA-CPB^-CTE^-EGFP (F/T) was significantly higher in G1 and G2 groups at T0-T5 as compared to G3 (*p*<0.001, *p*< 0.001, *p*<0.001, *p*<0.001 *p*<0.01 and *p*<0.001, respectively) (Fig 2F).

The levels of TNF-α production in PBMCs in response to *L*. *infantum* (F/T) were significantly higher in G1 than in G2 and G3 at T3 and T5 (*p*<0.05 and *p*<0.01, respectively) and only at T5 in G2 (*p* < 0.05, Fig 2G). We also observed significantly higher levels of TNF-α following stimulation with *L*. *tarentolae* A2-CPA-CPB^-CTE^-EGFP (F/T) in G1 at T1, T2 and T5 (*p*<0.01, *p*<0.05 and *p*<0.05, respectively) and for G2 only at T2 (*p*<0.05) in compared to G3 (Fig 2H).

Altogether, the levels of IFN-γ and TNF-α significantly increased in vaccinated group (G1) whereas levels of IL-10 significantly decreased in comparison to the control group (G3). Moreover, we analyzed the correlation between the IFN-γ and IgG2 at fourteen and seventeen months after challenge in all groups. Our results showed that G1 had the highest correlation between IFN-γ and IgG2 production for both periods (Spearman r = 0.99, *p*< 0.001) in comparison to the other groups as shown in S2 Fig.

### Delayed-type hypersensitivity response

Delayed type hypersensitivity (DTH) against *L*. *infantum* promastigotes was tested after 11 and 16 months post-challenge. All dogs developed DTH response as measured 11 months after infection (Fig 3A). The size of the indurations was determined 48 hours after administration of *L*. *infantum* antigens. The G1 group showed a significantly higher (*p<* 0.05) DTH response compared to G3 (Fig 3A). We also observed that 77% of dogs in G1 had an induration higher than 10 mm in comparison to G2 and G3 in which only 33% showed this pattern. Interestingly, at 16 months post-challenge, although G1 had higher DTH response (55% have more than 10 mm induration), there was no significant difference between these groups. Of note, one dog in the G1 and two dogs in G2 and G3 did not show any DTH response at 16 months post-challenge (Fig 3B). Overall, vaccinated group (G1) demonstrated a strong DTH response in comparison to the control group (G3).

**Fig 3:** Size of induration after injection of *L*. *infantum* stationary phase promastigotes in 0.4% phenol-saline to measure skin test reactivity. Data represent the individual delayed type of hypersensitivity responses in millimeter at months11 (A) and 16 (B) after infection. DTH reaction was determined by injecting intradermally in the inner aspect of the right hind leg with 0.1 ml of *L*. *infantum* in 0.4% phenol-saline antigen (3×10^8^ stationary phase promastigotes/ml). The left hind leg received only 0.1 ml 0.4% phenol saline solution. Data represent the increase of intradermal reaction performed 48 hrs after antigen injection. The values of the saline control were subtracted from the reaction due to the *Leishmania* antigen. Reactions ≥5mm were considered as positive.

### Low parasite density in vaccinated groups

Bone marrow is an important lymphoid organ in clinical analyses of canine visceral leishmaniasis. In the present study, the amount of *Leishmania* DNA (due to *L*. *infantum*) was detected by quantitative PCR in bone marrow samples at 18 months post-challenge.

As shown in Fig 4, dogs vaccinated with *L*. *tarentolae* A2-CPA-CPB^-CTE^-EGFP (G1) exhibited significantly lower parasite numbers in bone marrow when compared to the PBS group (G3) (*p<*0.05), whereas no significant difference was observed between G2 and G3 (*p>*0.05).

**Fig 4:** Determination of parasite quantities in the bone marrow of vaccinated and control groups. Number of parasites was determined by real-time PCR in bone marrow samples (BM) at 18 months post-infection. Results were calculated by means of an absolute method, by comparison of Ct values with those from a standard curve constructed from 10-fold dilutions of *L*. *infantum* DNA extracted from cultured parasites, from 1×10^6^ to 0.1 parasite equivalents/ml. Data are represented as number of parasites/μg of bone marrow DNA. The asterisks indicate that differences are statistically significant (*p* < 0.05). n.s. denoted as non significant.

### Cytological and immunocytochemical findings

Quantified amastigote density in Fine Needle Aspiration (FNA) and ICC smears for *Leishmania* were classified by two independent observers. The density of amastigotes in the G1 (vaccinated group) was grade I and II. Respectively, three and six cases of G1 showed grade I and grade II cytologically as well as immunocytochemically (Table 1). The density of amastigotes in the G2 and G3 was varying from grade I to IV. Two cases of both G2 and G3 groups had grade I, also four cases of G2 and two cases of G3 was verified as grade II. One case of G2 and two cases of G3 showed grade III. Severe parasite loading (grade IV) was seen in one case of G2 and three cases of G3. Cytologically and immunocytochemically, the density of amastigotes in G1 was lower than in G2 and G3 as shown in Table 1 and Fig 5. Cytologically, there was no dog with grade III and IV in group G1 as compared to G2 and G3 (2 dogs in G2 and 5 dogs in G3 with grade III and IV). Our observations indicate that group G3 had the highest number of dogs with grade III and IV (*p*<0.05).

**Fig 5:** Immunocytochemical (ICC) staining of bone marrow with different infection grades (grades I, II, III and severe infection as grade IV) in dogs of different groups. Panels A and B show infection with grade I and II belonging to G1; panels C and D infection with grades II and III belonging to G2; panels E and F, infection with grades III and IV belonging to G3. Intracytoplasmic leishman bodies (arrow headed), free leishman bodies (arrows), magnification X200.

### Clinical status and laboratory findings

Different criteria were used for dividing the dogs into three categories, including sub patent (only positive for bone marrow PCR), asymptomatic (bone marrow PCR positive, spleen culture positive with minor biochemistry abnormality and minor weight loss) and symptomatic (bone marrow PCR positive, spleen culture positive, intensive weight loss and strong clinical biochemistry abnormality). The main clinical features presented by dogs are summarized in Table 3. Clinical signs of VL appeared at the earlier stage in dogs of control group (G3) as compared to the vaccinated dogs in G1. In addition, 56% of dogs in the control group were symptomatic whereas 33% of vaccinated group (G1) and 34% of G2 were symptomatic. One animal in each of G2 and G3 presented a progressive form of VL signs and died, whereas none died in G1. The evaluation of different biochemical parameters related to protein alterations showed a significant difference in the AST, Alb, ALP, Urea, creatinine and total proteins concentration between G1 and G3 (*p*< 0.05). Between G2 and G3, we observed a significant increase in the levels of AST and total protein in the G3. There were no significant differences in respect to the ALT levels between groups. Altogether, the clinical findings showed that control group (G3) had the highest symptomatic dogs in comparison to G1 and G2 groups.

**Table 3:** Clinical status of dogs and percentage of each group within each category.

	Bone marrow PCR^a^	Spleen culture ^a^	Clinical biochemistry abnormality	Weight lost	G1	G2	G3
**Sub patent**	+	-	None	None	34%	22%	11%
**Asymptomatic**	+	-	+^b^	Minor^c^	33%	44%	33%
**Symptomatic**	+	+	++^b^	Intensive^d^	33%	34%	56%

^a^ *L*. *infantum* was detected by PCR in the bone marrow aspirates or by the culture of spleen collected 18 and 20 months post-infection, respectively.

+^b^ = lower than 3 biochemical parameters with abnormalities

++^b^ = more than 3 biochemical parameters with abnormalities

Minor^c^ = weight loss less than 2 Kg

Intensive^d^ = weight loss more than 3 Kg

## Discussion

Here, we vaccinated dogs with a live-vectored vaccine against VL using a non-pathogenic protozoan parasite, *L*. *tarentolae*, expressing the *L*. *donovani* A2 antigen along with CPA and CPB cysteine proteinases and tested its immunogenicity and protective potential against infectious challenge. Our previous study demonstrated that vaccination of dogs with cysteine proteinases type I and II (CPB and CPA) elicited an increased expression of IFN-γ mRNA and a strong parasite-specific Th1 response and conferred protection against parasite challenge [29]. Fernandes *et al*. also showed that immunization with rA2 antigen was immunogenic and induced partial protection in dogs, associated with increased IFN-γ and low IL-10 levels detectable in vaccinated animals before and after challenge [23].

In this study, we have evaluated both cellular and humoral immunity associated with post-vaccination protection against *L*. *infantum*. We demonstrated that vaccination with *L*. *tarentolae* A2-CPA-CPB^-CTE^-EGFP induced an antibody response that reacted with *L*. *infantum*. There is some experimental evidence that antibody production may have some roles in protection against VL. It has indeed been reported that antibodies induced by vaccination interfered not only with the parasite survival and multiplication but also with binding and/or internalization of promastigotes by macrophages [39]. In our study, the levels of IgG1 increased in response to *L*. *infantum* (F/T) in all groups after infection but in the PBS control group (G3), the levels of IgG1 were significantly higher than in groups G1 and G2 immunized with *L*. *tarentolae* A2-CPA-CPB^-CTE^-EGFP and *L*. *tarentolae* WT, respectively. The post-infection level of IgG2 increased in all groups but group G2 demonstrated the highest level of IgG2. The level of IgG2 in vaccinated group (G1) was significantly higher than the PBS group only at seventeen months post-challenge. There are several studies demonstrating an association of high IgG2 production with asymptomatic infections and elevated IgG1 levels with disease [39, 40]. Here, we showed that the levels of *Leishmania*-specific IgG2 were higher than those of *Leishmania*-specific IgG1 antibody in dogs vaccinated with recombinant *L*. *tarentolae* A2-CPA-CPB^-CTE^-EGFP. In contrast, levels of the IgG1 subclass were higher than IgG2 in dogs that received PBS only, in agreement with some previous reports [41–43]. Although all experimentally infected dogs in our study developed anti-*L*. *infantum* antibody responses, there is, however, some controversy over the association between canine IgG subclass ratio and protective cellular immune responses in canine visceral leishmaniasis [43–48]. It has been suggested that the IgG2 / IgG1 ratio in dogs infected with *L*. *infantum* is an alternative measure of Th1 ⁄ Th2 polarization of the immune response [29, 49]. It has been reported that IgG2 ⁄ IgG1 ratio in vaccinated and protected dogs is >1 whereas the ratio of <1 is due to canine visceral leishmaniasis (CVL) with progression towards overt disease [50]. In this study, the IgG2 ⁄ IgG1 ratio at T5 in all vaccinated groups (G1, 100%) was more than 1 in contrast to G2 (77%) and G3 (55%).

Here, we found that the levels of IFN-γ increased after infection in the vaccinated group (G1) in comparison to the PBS group (G3). Higher levels of IFN-γ were observed at two, fourteen and seventeen months after challenge. It is worth mentioning that at fourteen and seventeen months after challenge in G1, the peak production of IFN-γ in response to vaccination occurred concurrently with the significant elevation of IgG2 and this correlation was higher than in the other groups. This suggests that the recombinant *L*. *tarentolae* A2-CPA-CPB^-CTE^-EGFP polarizes the immune system towards a Th1 response and that high levels of IFN-γ can stimulate macrophages to kill *Leishmania* amastigotes. These results are in agreement with previous studies showing that the main effector mechanism involved in protective immune response of dogs infected with *L*. *infantum* is the activation of macrophages by IFN-γ and TNF-α to kill intracellular amastigotes via the nitric oxide pathway [51]. It has been shown that NO production and anti-leishmanial activity were also detected in a canine macrophage cell line infected with *L*. *infantum* after incubation with IFN-γ, TNF-α and IL-2 [52] as well as in macrophages from dogs immunized with killed *L*. *infantum* promastigotes [53]. IFN-γ was seen to increase and correlate with protection in vaccinated dogs [54–56]. A large number of studies using putative protective antigens or attenuated parasites in mice have shown that protection against progressive visceral infection involves high expression of IFN-γ and decreased expression of IL-10 [57–59]. In dogs, low parasite burdens of *L*. *chagasi* in lymph nodes were also associated with high expression of IFN-γ and TNF-α [60]. Also, recent studies in dogs showed that live attenuated *L*. *donovani* with the centrin gene deleted (LdCen−/−) were capable of inducing protection against an infectious *L*. *infantum* challenge. This protection was associated with significantly higher production of IFN-γ, IL-12/IL-23p40 and TNF-α that skewed type 1 immune response hence contributing to a remarkable reduction in bone marrow parasite load [55, 56]. The elevated expression of IFN-γ during severe disease has also been described in patients with active VL [61, 62]. TNF-α has also been shown to play a protective role by synergizing with IFN-γ in mediating parasite killing [63]. In the present study, levels of TNF-α were significantly higher in the vaccinated group G1 against *L*. *infantum* F/T antigen during T1, T3 and T5 periods.

Here, we found that the IL-10 levels in the vaccinated group G1 were lower in comparison to the PBS group during the periods T2-T5. Our results showed that recombinant *L*. *tarentolae* A2-CPA-CPB^-CTE^-EGFP changes the immune profile to Th1. Previous studies showed that IL-10 is related to progressive disease in human visceral leishmaniasis [62] and plays a role in susceptibility to VL in hamsters and murine models [64]. Other studies also showed that high IL-10 expression was associated with increase in parasitic loads and progression of the disease [65, 66]. Also, increased levels of IL-10 mRNA were reported in PBMCs from control infected dogs after challenge with *L*. *infantum* [29]. In human *L*. *chagasi* infection, IL-10 production has been correlated with pathology [67]. Taken together these reports are in agreement with our findings. IFN-γ to IL-10 ratio is another relevant indicator of successful immunization [38]. The IFN-γ/IL-10 ratio in G1 stimulated with *L*. *infantum* F/T increased significantly after challenge during 11 to 17 months in comparison to the PBS group. Furthermore, the IFN-γ/IL-10 ratio against recombinant *L*. *tarentolae* A2-CPA-CPB^-CTE^-EGFP (F/T) in G1 and G2 was significantly higher than in G3 at all tested time intervals post-challenge.

Skin delayed-type hypersensitivity (DTH) response has been used as another indicator of the immunogenicity of an antigen immunization, measured by the presence of a specific cellular type of immune reaction [68–70]. Positive DTH response is a marker of a type 1 immune response and has been used to assess the immunogenicity of candidate vaccine antigens against leishmaniasis [68, 70, 71]. Our results demonstrated a DTH response in all dogs after infection but in vaccinated group (G1) this response was stronger both at 11 and 16 months post-challenge. It has been shown previously that in naturally infected groups, those that were asymptomatic and did not progress to active visceral disease had a stronger DTH response compared to dogs that progressed to an active VL [72, 73].

Parasite density in the bone marrow and spleen was the most reliable marker to explore the clinical status of CVL [74]. It has been shown that bone marrow parasite density could act as a factor of major phenotypic changes in peripheral blood leukocytes in canine visceral leishmaniasis. Also, it was reported that dogs displaying higher bone marrow parasite density are more likely to develop severe CVL [56, 75]. In this study, parasite density in bone marrow of all dogs was evaluated by reliable methods including direct detection (cytology and ICC) and real time PCR. Recent findings showed a high sensitivity in detection of *L*. *infantum* DNA by real-time PCR. These results indicate the usefulness of this method for quantification of *Leishmania* DNA [76, 77]. The results of direct detection particularly ICC showed the highest density of amastigotes in G3, followed by G2. These findings are in agreement with other obtained results. High sensitivity and specificity of ICC in amastigote detection has been reported recently [35]. The vaccinated group (G1) showing partial protection had significantly the lowest quantity of parasites compared to the PBS group (G3). In group G2, almost all dogs (with the exception of two) showed lower quantity of parasites in comparison to G3. Our results indicate that although immunization with recombinant *L*. *tarentolae* A2-CPA-CPB^-CTE^-EGFP (G1) induced significantly higher immune response in comparison to the control group (G3), G2 that was immunized with wild type *L*. *tarentolae* demonstrated a similar clinical status as G1 at 20 months post-infection.

In conclusion, our study supports that live vaccination with recombinant *L*. *tarentolae* A2-CPA-CPB^-CTE^-EGFP as prime/boost vaccine is shown to be safe and immunogenic in uninfected, unexposed outbreed dogs. After experimental infection with promastigotes, all dogs progressed from subpatent infection to asymptomatic and finally to symptomatic infection. The vaccinated group (G1) had the highest percentage of subpatent stage (34% in comparison to 22% in G2 and 11% in G3) and lowest percentage of symptomatic stage (33% in comparison to 56% in G3). It is worth mentioning that the full picture of the *in vivo* response in dogs is very complex and hardly can correlate individual markers with absolute resistance to disease. Therefore, it is important to take all parameters into account to conclude that there is protection. In our study, the experimental challenge with high levels of metacyclic parasites may have underestimated the vaccine efficacy results. Although it is a matter of speculation, if a more relevant (smaller dose, intradermal inoculation) challenge were used, higher levels of protection could be observed. Our results indicate that although vaccination with *L*. *tarentolae* A2-CPA-CPB^-CTE^EGFP may not prevent the disease in all cases, it could render the disease development slower and milder (considering clinical observation and weight lost) in vaccinated groups. If the development of the disease can be slowed down in cases where it cannot be prevented, this could favor early treatment with better longer-term survival. The work presented here is among the first line of research using vectored based vaccination in dog models and could act as a platform for future studies in large animals. Using this strategy, it would be possible to consider only one time immunization by further improving our live vaccine regimen to enhance protective and long-term immune responses, may be by using some immune-potentiators such as CpG-ODN. In future experiments, we could also include to our live vaccine regiment the immunogenic component of salivary gland of sand fly. Recently, we showed that a combination of recombinant *L*. *tarentola*e with a sand fly salivary antigen (PpSP15) of *Ph*. *papatasi* has elicited strong protective immune responses against cutaneous leishmaniasis in both resistance and susceptible mice against *L*. *major* infection [78].

## Supporting Information

S1 Fig Experimental setup and timelines. Three groups of dogs were allocated for this experiment. According to their weight, sex and age dogs were divided in three groups (each including 10 dogs) named as G1, G2 and G3. They have immunized two times with three weeks intervals. Before challenge, both humoral and cellular immune responses were assessed. At different time periods after infectious challenge with *L*. *infantum*, besides the immune response evaluation, DTH, parasite burden as well as cytology and immunohistochemistry were carried out.
(TIF)

S2 Fig Correlation between IFN-γ and IgG2 at two different time periods. Increased levels of IFN-γ production had the highest correlation with the level of IgG2 (Spearman r = 0.99, P<0.001) at 14 (panel A) and 17 (panel B) months after challenge in G1 as compared with G2 and G3. At each time period, r^2^ for each group was determined as shown in the S2 Fig.
(TIF)
